The article "HHLA2 Used as a Potential Prognostic and Immunological Biomarker and Correlated with Tumor Microenvironment in Pan-Cancer" was retracted in 2024. Reasons: signs of a paper mill; suspected computer-generated content; unreliable results or conclusions; concerns about the data.

# HHLA2 Used as a Potential Prognostic and Immunological Biomarker and Correlated with Tumor Microenvironment in Pan-Cancer

**DOI:** 10.1155/2022/3924400

**Published:** 2022-02-23

**Authors:** Zeng Yang, Diao Xu, Xiao Ye, Xuehua Lin, Min Zhang, Yan Su, Qun Xie, Wenjun Ni

**Affiliations:** Department of Urology, Zhuhai People's Hospital (Zhuhai Hospital Affiliated with Jinan University), Zhuhai, China

## Abstract

**Background:**

The role of HERV–H LTR-associating 2 (HHLA2) in cancer remains still unclear. This study analyzed the correlation between the prognosis and immune infiltrate function of HHLA2 in pan-cancers.

**Methods:**

HHLA2 expression in pan-cancers was analyzed using the databases of TCGA, GTEx, TIMER, GEPIA, UALCAN, and GSEA databases. Multiple bioinformatic methods were used to investigate the correlation of HHLA2 expression with survival, pathological stage, tumor mutation burden (TMB), microsatellite instability (MSI), tumor microenvironment (TME), immune cell infiltration, and immune checkpoint gene (ICG), and gene functional enrichment was performed by Gene Set Enrichment Analysis (GSEA) and Gene Set Variation Analysis (GSVA).

**Results:**

HHLA2 was aberrantly expressed and was strongly correlated with positive or negative prognosis in multiple human cancers, which revealed that HHLA2 might play a vital role during cancer formation and development. Kaplan–Meier (KM) curves across cancers revealed that HHLA2 expression was correlated with overall survival (OS) in eight cancers, disease-specific survival (DSS) in seven cancers, disease-free interval (DFI) in four cancers, and progression-free interval (PFI) in nine cancers. Furthermore, HHLA2 expression was positively correlated with TMB in 6 cancer types and negatively associated with TMB in 7 cancer types, respectively. The former included ESCA, HNSC, KIRP, PAAD, PRAD, and PCPG; the latter contained COAD, LGG, LUAD, LUSC, THYM, THCA, and UCEC. Additionally, we found HHLA2 expression was negatively related to MSI in ACC, COAD, PAAD, and UCEC. More importantly, HHLA2 expression was remarkably correlated with the degree of tumor-infiltrating immune in many cancers, including B cells, CD4+ T cells, CD8+ T cells, neutrophils, macrophages, and dendritic cells and strongly associated with immune checkpoint genes in 13 tumor types. Furthermore, KEGG pathway analyses indicated that HHLA2 could potentially impact cancer etiology or pathogenesis by functioning in amino sugar and nucleotide sugar metabolism, cytosolic DNA sensing pathway, and peroxisome pathways. Meanwhile, GSVA analysis results all indicate that HHLA2 was correlated with TSC/mTOR, RTK, RAS/MAPK, PI3K/AKT, EMT, DNA Damage Response, Cell Cycle, and Apoptosis pathways in various cancers.

The article "HHLA2 Used as a Potential Prognostic and Immunological Biomarker and Correlated with Tumor Microenvironment in Pan-Cancer" was retracted in 2024. Reasons: signs of a paper mill; suspected computer-generated content; unreliable results or conclusions; concerns about the data.

**Conclusion:**

HHLA2 can function as a prognostic biomarker and correlate with tumor immunity in human pan-cancer due to its important role in tumorigenesis and immune infiltration, which provides new insight into developing new targeted treatments in cancers.

## 1. Introduction

Cancer is one of the major obstacles threatening the quality of life in the world. Over the past few decades, the morbidity and mortality of malignant tumors globally have imposed substantial health and economic burden on society [1]. In recent years, specific gene targeted therapy and immunotherapy have been counted as exhilarating therapeutic strategies, but they have not received satisfactory outcomes yet [2]. Although substantial advances in therapies and medical technologies improve the rate of some clinical success, the prognosis and survival rate for patients with cancer are unsatisfactory, which is attributed to drug resistance, the complexity of the occurrence, development of cancer, and prognosis [3]. As we all know, tumorigenesis is a complicated and multistep process. Several studies have reported that the tumor microenvironment (TME), comprising a large proportion of infiltrating immune cells, plays an important role in oncogene activation and the production of abnormal proteins and stress signals in human cancers [4, 5]. Therefore, it is necessary to explore the novel sensitive tumor biomarkers and the mechanism of their interaction with tumors in the immunotherapy of cancer [6]. Human endogenous retrovirus-H long terminal repeat-associating protein 2 (HHLA2), a newly discovered B7 family member, is analogous to PD-L1, PD-L2, and B7-H3 and encodes a protein-ligand found on the surface of monocytes [7]. The encoded protein is thought to be involved in tumor immune evasion by binding to a receptor on T lymphocytes and inhibiting the proliferation and cytokine production of CD4+ and CD8+ T cells. TMIGD2, a single-pass type I membrane protein containing one immunoglobulin-like domain, is the only evidenced receptor of HHLA2 [8]. Therefore, HHLA2 may also have a potential role in tumor angiogenesis. Janakiram et al. [9] demonstrated that HHLA2 is widely expressed in a large proportion of cancer samples such as breast cancer, colon cancer, and prostate cancer. In recent years, studies have shown that HHLA2 participates in the growth and development of a variety of cancers [7, 10, 11]. However, to date, the expression pattern, prognostic significance, and biological function of HHLA2 in cancer have not been elucidated fully. Given the complexity of tumorigenesis, analyzing the pan-cancer expression of the genes we are interested in and identifying certain functional and pathway genes correlated with various human malignancies, including clinical prognosis and potential molecular mechanisms, are very significant.

The article "HHLA2 Used as a Potential Prognostic and Immunological Biomarker and Correlated with Tumor Microenvironment in Pan-Cancer" was retracted in 2024. Reasons: signs of a paper mill; suspected computer-generated content; unreliable results or conclusions; concerns about the data.

In this study, taking advantage of the gene expression data and clinical information from TCGA and other tumor research databases was the first time to access the expression level and prognostic value of HHLA2 pan-cancer analysis. We then explored the potential relationships between HHLA2 expression and tumor microenvironment (TME), microsatellite instability (MSI), tumor mutational burden (TMB), and immune checkpoints for different types of the tumor using correlation analysis. Meanwhile, Gene Set Enrichment Analysis (GSEA) and Gene Set Variation Analysis (GSVA) were employed to illustrate the potential biological function of HHLA2 in many cancers. The results of the present study reveal that HHLA2 is associated with tumorigenesis and tumor microenvironment and might be used as a novel prognostic biomarker in pan-cancer.

## 2. Materials and Methods

### 2.1. Raw Data Acquisition and Processing

UALCAN software (https://ualcan.path.uab.edu/analysis.html), an integrated data-mining platform to facilitate the comprehensive analysis of cancer transcriptome, uses TCGA RNA-sequencing and patients' clinical data from 33 types of human malignancies, including several metastatic tumors [12]. Using UALCAN, it is possible to explore the pan-cancer expression pattern of the HHLA2 gene in tumor tissues and tumor samples and normal samples from TCGA database. TCGA (The Cancer Genome Atlas) had profiled and analyzed a large collection of clinical and molecular data from 33 types of cancers [13]. The GTEx program (https://gtexportal.org/), a tissue bank and data resource, has aggregated more than 7,000 samples, covering 53 normal human tissues [14]. UCSC Xena Shiny (https://shiny.hiplot.com.cn/ucsc-xena-shiny/) was used to obtain 33 cancer-related level 3 RNA-sequencing data sets and their associated clinical data. Given that TCGA included fewer normal samples, we integrated normal tissue data from GTEx with tumor tissue data from TCGA to analyze the expression differences of HHLA2. The TIMER database (https://cistrome.shinyapps.io/timer/) is a web resource with 10,897 samples from various cancer types, which is used to assess the clinical impact of the infiltration of immune cells on different cancer types via the TIMER algorithm [15]. Additionally, we took advantage of the TIMER website to analyze the differential expression of HHLA2 between tumor tissues and normal tissues for diverse cancers.

### 2.2. Survival and Prognosis

Survival and clinical data of different cancers were extracted from TCGA. We then selected four indicators, including overall survival (OS), disease-specific survival (DSS), disease-free interval (DFI), and progression-free interval (PFI), to study the association of HHLA2 expression with the prognosis of patients in 33 kinds of cancers via forest plots in UCSC Xena Shiny (https://shiny.hiplot.com.cn/ucsc-xena-shiny/) and Kaplan–Meier curves using Kaplan–Meier Plotter (https://kmplot.com/analysis/). The forest plots and Kaplan–Meier (KM) curves were used for survival analyses (*p* < 0.05).

The article "HHLA2 Used as a Potential Prognostic and Immunological Biomarker and Correlated with Tumor Microenvironment in Pan-Cancer" was retracted in 2024. Reasons: signs of a paper mill; suspected computer-generated content; unreliable results or conclusions; concerns about the data.

### 2.3. Correlation of HHLA2 Expression with Immune Checkpoints, MSI, and TMB

TMB is a quantifiable and profound biomarker that is associated with overall survival (OS) after immune checkpoint inhibitor therapy for various cancers. Tumor mutational burden (TMB) refers to the total amount of mutations per DNA megabases, including insertions, base substitutions, or deletions across bases [16, 17]. Microsatellite instability (MSI), an important clinical tumor marker associated with DNA MMR defects, referred to the occurrence of new microsatellite alleles at a microsatellite locus in tumors [18]. The connections between HHLA2 expression and TMB and MSI were evaluated by utilizing Spearman's correlation analysis. Additionally, the relationship between HHLA2 and the immune checkpoints CD274, CTLA4, HAVCR2, LAG3, PDCD1, PDCD1LG2, TIGIT, and SIGLEC15 was analyzed based on TCGA data. Assistant for clinical bioinformatics (https://www.aclbi.com/) was used to explore to the correlation of HHLA2 expression with immune checkpoints, MSI, and TMB.

### 2.4. Immune Correlation Analysis

Tumor Immune Evaluation Resource is a free and publicly accessible database, which is used to detect the clinical impact of the infiltration of immune cells on different cancer types. In this study, six types of immune cells were assessed among different types of cancers, including B cells, CD4+ T cells, CD8+ T cells, neutrophils, macrophages, and dendritic cells. The UCSC Xena Shiny was used to investigate correlation analysis.

### 2.5. Gene Set Enrichment Analysis

Gene Set Enrichment Analysis (GSEA) and the Gene Set Variation Analysis (GSVA) were conducted to investigate the biological functions of HHLA2 in various cancers. Taking advantage of JAVA (https://software.broadinstitute.org/gsea/index.jsp), Gene Set Enrichment Analysis (GSEA) was employed to assess the biological functions of HHLA2 in tumors based on the “Molecular Signatures Database” of c2.cp.kegg.v7.1.symbols. We classified the patients into two groups based on their risk values. Gene sets with NOM *p* < 0.05 and FDR *q* < 0.25 were counted as significant enrichment results [19]. GSCA (Gene Set Cancer Analysis, https://bioinfo.life.hust.edu.cn/GSCA/#/) was chosen to study the correlation between GSVA score and pathway activity. GSVA score represents the variation of gene set activity over a specific cancer's sample population in an unsupervised manner. The pathway GSCA included are TSC/mTOR, RTK, RAS/MAPK, PI3K/AKT, EMT, DNA Damage Response, Cell Cycle, and Apoptosis pathways.

The article "HHLA2 Used as a Potential Prognostic and Immunological Biomarker and Correlated with Tumor Microenvironment in Pan-Cancer" was retracted in 2024. Reasons: signs of a paper mill; suspected computer-generated content; unreliable results or conclusions; concerns about the data.

### 2.6. Statistical Analysis

The Wilcoxon test was used to evaluate the differences in HHLA2 expression levels between tumor and normal tissues. Survival curves were generated using the Kaplan–Meier plotter database by the univariate Cox regression. Spearman's correlation analysis was calculated between HHLA2 expression and TMB, MSI, and immune checkpoint marker level. *p* < 0.05 was regarded as significant for all statistical analyses.

## 3. Results

### 3.1. Pan-Cancer Expression Analysis of HHLA2

Using UALCAN software, HHLA2 was the significant expression in tumor samples, including CHOL, COAD, ESCA, HNSC, KIRC, KIRP, LIHC, LUAD, LUSC, PAAD, STAD, READ, and UCEC (Figure 1(a)). HHLA2 expression was significant differences between tumor samples and normal samples in 12 malignancies, including COAD, ESCA, KICH, KIRC, KIRP, LUAD, LUSC, PAAD, READ, SARC, STAD, and UCEC (Figure 1(b)). We also compared the HHLA2 expression between the adjacent normal and cancer tissues by merging the data from TCGA and GTEx databases using UCSC Xena Shiny. As graphed in Figure 1(c), HHLA2 mRNA levels also increased significantly in breast invasive carcinoma (BRCA), CHOL, COAD, esophageal carcinoma (ESCA), glioblastoma multiforme (GBM), HNSC, KICH, KIRC, KIRP, acute myeloid leukemia (LAML), brain lower-grade glioma (LGG), lung adenocarcinoma (LUAD), LUSC, pancreatic adenocarcinoma (PAAD), pheochromocytoma and paraganglioma (PCPG), READ, stomach adenocarcinoma (STAD), thyroid carcinoma (THCA), uterine corpus endometrial carcinoma (UCEC), and uterine carcinosarcoma (UCS). As shown in Figure 1(d), the outcomes of HHLA2 expression from the TIMER database, in most cancers of cholangiocarcinoma (CHOL), colon adenocarcinoma (COAD), head and neck squamous cell carcinoma (HNSC), kidney chromophobe (KICH), kidney renal clear cell carcinoma (KIRC), kidney renal papillary cell carcinoma (KIRP), lung squamous cell carcinoma (LUSC), prostate adenocarcinoma (PRAD), rectum adenocarcinoma (READ), and uterine corpus endometrial carcinoma (UCEC) is higher than their adjacent normal tissues (*p* < 0.05). These findings indicate the differences in the expression of HHLA2 in human pan-cancer.

### 3.2. Prognostic Value of HHLA2 in Cancers

We investigated the association between the HHLA2 expression and the prognosis of survival correlation analyses in 33 cancers, including overall survival (OS), disease-free survival (DSS), disease-free interval (DFI), and progression-free interval (PFI). According to the Cox proportional hazards model analysis, the results suggested that HHLA2 expression positively correlated with OS in patients with KIRC (*p* < 0.001), READ (*p* = 0.014), and (SKCM) (*p* = 0.016) and negatively with OS in PRAD (*p* = 0.0043) (Figure 2(a)). Moreover, we analyzed the DSS data (Figure 2(b)) and suggested positively associations between HHLA2 expression and prognosis in patients with KIRC (*p* < 0.001), (SKCM) (*p* = 0.019), and THYM (*p* = 0.020); however, the HHLA2 expression exhibited the opposite relationship in PAAD (0.020). Regarding associations between HHLA2 expression and DFI, we found that HHLA2 expression affected patients' DFI in two cancer types, including PAAD (*p* = 0.016) and ESCA (*p* = 0.049) (Figure 2(c)). Furthermore, the forest plots showed that the expression impacted PFI in KIRC (*p* < 0.001) and PCPG (*p* = 0.019), while negative expression was associated with poor PFI in PAAD (*p* = 0.033) (Figure 2(d)). Moreover, Kaplan–Meier OS curves exhibited that an upregulated HHLA2 expression indicated poor prognosis in KICH (*p* = 0.0033), LAML (*p* = 0.046), LIHC (*p* = 0.0021), and PAAD (*p* = 0.0027), while low HHLA2 expression was related to poor OS in BLCA (*p* = 0.038), KIRC (*p* < 0.001), READ (*p* < 0.001), and SKCM (*p* = 0.0052) (Figure 3). Kaplan–Meier analysis indicated that the increased HHLA2 expression was remarkably associated with poor DSS in patients with KICH (*p* = 0.0032), PAAD (*p* = 0.0045), and UCEC (*p* = 0.034), while low HHLA2 expression was associated with poor DSS in KIRC (*p* < 0.0001), KIRP (*p* = 0.016), LUAD (*p* = 0.044), and SKCM (*p* = 0.011) (Figure 4). Kaplan–Meier analysis also indicated that high HHLA2 expression corresponded with poor DFI in patients with KIRC (*p* = 0.022), PAAD (*p* = 0.0063), while low HHLA2 expression was connected with poor DFI in COAD (*p* = 0.028) and ESCA (*p* = 0.0011) (Figure 5). Meanwhile, Kaplan–Meier analysis revealed that high HHLA2 expression was also linked with worse PFI in individuals with ESCA (*p* = 0.011), KICH (*p* = 0.016), and LIHC (*p* = 0.041), while low HHLA2 expression was related to poor PFI in BRCA (*p* = 0.037), CESC (*p* = 0.03), COAD (*p* = 0.023), HNSC (*p* = 0.042), KIRC (*p* < 0.0001), and KIRP (*p* = 0.03) (Figure 6). Above all, these results demonstrate the expression of HHLA2 influenced the prognosis of multiple cancers, whether OS, DFI, or PFI.

The article "HHLA2 Used as a Potential Prognostic and Immunological Biomarker and Correlated with Tumor Microenvironment in Pan-Cancer" was retracted in 2024. Reasons: signs of a paper mill; suspected computer-generated content; unreliable results or conclusions; concerns about the data.

### 3.3. Pan-Cancer Analysis of the Correlation between HHLA2 Expression and Clinicopathology

To assess the association between the HHLA2 expression and clinicopathological stages in multiple cancers, we investigated the HHLA2 expression in stages I, II, III, and IV. The results from TCGA database revealed that HHLA2 expression was significantly upregulated in advanced tumors in BRCA, ESCA, HNSC, LUSC, and UCS (Figure 7). These results indicated that HHLA2 expression was in correlation with the tumor stages of patients.

### 3.4. Relationship between HHLA2 Expression and TMB and MSI in Cancers

In the study, the relationship analysis of results between HHLA2 expression and TMB revealed that HHLA2 expression had positive relevance to TMB in ESCA, HNSC, KIRP, PAAD, PRAD, and PCPG. On the contrary, HHLA2 expression was negatively associated with TMB in COAD, LGG, LUAD, LUSC, THYM, THCA, and UCEC (Figure 8(a)). According to the results of the correlation of HHLA2 expression with MSI in human pan-cancer. We found HHLA2 expression was negatively corrected with MSI in ACC, COAD, PAAD, and UCEC (Figure 8(b)). These results indicated that HHLA2 expression was related to immunity in different types of cancer.

### 3.5. Pan-Cancer Analysis of the HHLA2 Expression and Immune Cell Infiltration and Immune Checkpoint

We used UCSC Xena Shiny to conduct a pan-cancer analysis of the correlation of HHLA2 expression with the immune cell infiltration level based on the TIMER database. We found that the HHLA2 expression was significantly linked with lots of infiltrating immune cells: B cells in 20 types of cancer, CD4+ T cells in 12 types of cancer, CD8+ T cells in 13 types of cancer, macrophages in 13 types of cancer, neutrophils in 12 types of cancer, and DCs in 15 types of cancer (Figure 9). Subsequently, we explored the association between HHLA2 expression and eight common immune checkpoint genes to examine whether HHLA2 could be a candidate as an underlying target for immune therapy in cancer. Interestingly, HHLA2 expression was correlated with five immune checkpoint genes in six tumors including DLBC, KIRP, LUAD, LUSC, SARC, and TGCT; was connected with six immune checkpoint genes in three tumors including GBM, KIRC, and THCA; was associated with seven immune checkpoint genes in three tumors including BLCA, BRCA, and LIHC; and was related to seven immune checkpoint genes in SKCM (Figure 10, Supplementary Table9). Collectively, these results show that HHLA2 acts significantly in immune infiltration.

### 3.6. Predicted Functions of HHLA2 in Cancers

We conducted a GSEA to analyze which KEGG pathways were correlated with HHLA2 expression in pan-cancers. Then, we classified patients into the high- and low-expression groups based on HHLA2 expression of the median. The top one term of KEGG analysis with enrichment results of NOM *p* < 0.05 and FDR *q* < 0.25 was exhibited. KEGG pathway analyses exhibited that HHLA2 could potentially impact cancer etiology or pathogenesis in high HHLA2 expression groups, including Alzheimer's disease in BRCA; amino sugar and nucleotide sugar metabolism in COAD; and regulation of actin cytoskeleton in HNSC. In addition to high HHLA2 expression groups, our results demonstrated that HHLA2 also regulates many other pathways in low HHLA2 expression groups, such as those involved in steroid hormone biosynthesis in ACC; cytosolic DNA sensing pathway in LAML; amino sugar and nucleotide sugar metabolism in KIRC; histidine metabolism in PAAD; peroxisome in PRAD; and systemic lupus erythematosus in UCEC (Figure 11). Then, we also investigated the correlation between GSVA score and pathway activity to further explore the biological significance of HHLA2 expression in multiple cancers. Briefly, the GSVA score represents the integrated level of the expression of HHLA2 gene set, which is positively correlated with HHLA2 expression. We observed the relationship between HHLA2 expression and six pathway activities using Spearman's rank correlation coefficient. The complex interaction is visualized in the form of chord graph. We visualized the results at *p* < 0.05. As shown in Figure 12 and Supplementary Table 10, the HHLA2 expression correlated significantly positively with Apoptosis resting in BLCA, BRCA, KIRP, LIHC, and SKCM, but significantly negatively with Apoptosis activated in KIRC, LUAD, and TGCT. HHLA2 expression also correlated significantly positively with Cell Cycle in COAD, PRAD, and THYM, but significantly negatively with Cell Cycle in KIRC, LUAD, LUSC, TGCT, and UCEC. Furthermore, the HHLA2 expression correlated significantly positively with DNA Damage in BRCA, OV, and THYM but substantially negatively in KIRC, LGG, LUAD, PAAD, and TGCT, significantly positively with EMT in LIHC but markedly negatively in COAD, ESCA, HNSC, KIRC, LGG, OV, READ, and STAD, significantly positively with PI3KAKT in KIRC and LUAD, but considerably negatively in LGG, PRAD, significantly positively with RASMAPK resting in CHOL, HNSC, LGG, LUAD, LUSC, and TGCT, but remarkably negatively in LIHC, PRAD, and THYM, and significantly positively with RTK resting in ESCA, LUAD, PAAD, STAD, and TGCT, but considerably negatively in LIHC and PRAD, significantly positively with TSC/mTOR in KIRP and STAD but markedly negatively in BRCA and TGCT.

The article "HHLA2 Used as a Potential Prognostic and Immunological Biomarker and Correlated with Tumor Microenvironment in Pan-Cancer" was retracted in 2024. Reasons: signs of a paper mill; suspected computer-generated content; unreliable results or conclusions; concerns about the data.

## 4. Discussion

Pan-cancer analysis can play a useful role in revealing the similarities and differences in tumors, providing new insight into cancer prevention, the design of therapeutic targets, and novel tumor biomarkers [20–22]. Recently, many studies have provided a new perspective on the genome-wide analysis of the early diagnosis and the identification of sensitive biomarkers in human pan-cancer, including gene mutations, RNA alterations, driver genes, and copy number alterations [23–25]. HHLA2 (Human endogenous retrovirus-H long terminal repeat-associating protein) is a recently described immune checkpoint molecule as a member of the B7-CD28 family, plays a vital role in the regulation of the immune system, and also costimulates and cosuppresses T cell proliferation and function and the production of cytokines [8, 26]. B7.2 (CTLA-4), B7.1 (PD-1), and B7-H1 (PD-L1) play an important role in costimulatory or coinhibitory molecules of the B7 family in tumor immune regulation. HHLA2, as a member of the B7-CD28 family, can bind CD4 and CD8 T cells and antigen-presenting cells and exert both coinhibitory and costimulatory functions [27]. HHLA2 is abnormally expressed in various malignant tumors, and it has been linked to angiogenesis, tumor growth, and metastasis.

In this study, we first comprehensively analyzed HHLA2 using TCGA, GTEx, TIMER, and KEGG databases in the pan-cancer to extensively demonstrate the function of HHLA2 as it relates to various cancers. Bioinformatic analyses were conducted to identify the HHLA2 expression-related KEGG pathways. According to the analysis of results HHLA2 expression in various malignancies, we found that HHLA2 was expressed differently in numerous cancers, and most cancer types had a higher number of HHLA2 alternations. According to the Cox and KM survival analysis, we found that abnormal expression of HHLA2 served as a prognostic factor in some types of cancer. Furthermore, we observed that HHLA2 expression was closely associated with immune infiltration and immune checkpoint markers in multiple cancers. Therefore, this study's results significantly indicated that HHLA2 played an essential role in tumor immunity and might act as a potential biomarker. Kaplan–Meier survival analysis using TCGA data showed that abnormal HHLA2 expression might be associated with patients' prognosis and play important roles in the occurrence and progression of these cancers. These previous findings also demonstrated that high HHLA2 expression was linked to poor prognosis in cancer. In the present report, our results showed that high HHLA2 expression was correlated with poor OS in five tumors, including KICH, LAML, LIHC, and PAAD. Similarly, it was previously reported that HHLA2 expression was linked to shorter survival time in patients with clear cell renal cell carcinoma [7], gastric cancer [28], and hepatocellular carcinoma [29]. By contrast, high HHLA2 expression is predictive of a good prognosis in patients with BLCA, KIRC, READ, and SKCM. These findings clearly suggest that HHLA2 may be counted as a biomarker to predict the prognosis of various cancers.

The article "HHLA2 Used as a Potential Prognostic and Immunological Biomarker and Correlated with Tumor Microenvironment in Pan-Cancer" was retracted in 2024. Reasons: signs of a paper mill; suspected computer-generated content; unreliable results or conclusions; concerns about the data.

In recent years, the tumor microenvironment has been counted as a promising prognostic biomarker of cancers and provides guidance for immunotherapy selection in the context of precision medicine [30]. Immune cells composed of neutrophils, natural killer cells, macrophages, dendritic cells, B cells, and T cells play vital regulatory roles in TME and are an important part of the tumor microenvironment, which is regarded as the “seventh marker feature” of the tumor [31]. More and more evidences have demonstrated that the interaction between cancer cells and various tumor-infiltrating lymphocytes which is a key component of TME promotes immune escape of tumors and ultimately contributes to tumor progression. MSI is also correlated with clinical characteristics and prognosis and is a vital biologic in immune-checkpoint inhibitors (ICI) [32, 33], which results in TMB and higher numbers of tumor-infiltrating lymphocytes [34]. These all indicate that immune cells in TME play a crucial role in the progression of multiple cancers [35–38]. However, few studies show that HHLA2 plays in the immune microenvironment. According to this study results, we found that BRAP expression was positively related to 6 immune infiltrating cells (B cells, CD4+ T cells, CD8+ T cells, dendritic cells, macrophages, and neutrophils). Furthermore, we found the coexpression of HHLA2 with eight immune checkpoint markers across cancers, specifically in BLCA, BRCA, LIHC, DLBC, KIRP, LUAD, LUSC, SARC, SKCM, TGCT, and THYM. The novel results of the correlation between HHLA2 expression and immune checkpoint markers implied that HHLA2 might recruit and regulate infiltrating immune cells to inhibit or promote the progression of cancers, which strongly reveals that the important role of HHLA2 in cancer immunity. Our study demonstrated that HHLA2 expression is correlated with TMB in 13 cancer types such as ESCA, HNSC, KIRP, PAAD, PRAD, and PCPG with MSI 13 cancer types including ACC, COAD, PAAD, and UCEC. Based on both previous studies and our own findings, this may indicate that high HHLA2 expression is positively correlated with high expression of TMB and MSI of cancer which provides a new reference for better prognosis of immunotherapy and response to ICI treatment. Therefore, our research sheds light on understanding the latent role of HHLA2 in tumor immunology and its use as a prognostic biomarker of cancers. Furthermore, KEGG pathway analyses indicated that HHLA2 could potentially impact cancer etiology or pathogenesis by functioning in amino sugar and nucleotide sugar metabolism, cytosolic DNA sensing pathway, and peroxisome pathways. Meanwhile, GSVA analysis results all indicate that HHLA2 was correlated with TSC/mTOR, RTK, RAS/MAPK, PI3K/AKT, EMT, DNA Damage Response, Cell Cycle, and Apoptosis pathways in various cancers. Therefore, our findings provided new insights into the development and treatment of HHLA2 in cancer.

The article "HHLA2 Used as a Potential Prognostic and Immunological Biomarker and Correlated with Tumor Microenvironment in Pan-Cancer" was retracted in 2024. Reasons: signs of a paper mill; suspected computer-generated content; unreliable results or conclusions; concerns about the data.

Nevertheless, this study still has several limitations. First, we only conducted a bioinformatic analysis of HHLA2 expression and patient survival across different databases, and thus, our results need to be approved in vitro and in vivo experiments in the future. Secondly, there is limited clinical data in public databases, and surgery, chemotherapy, and neoadjuvant therapy on clinical survival should also be taken into account. Finally, there is a need to conduct prognostic analysis of HHLA2 from multiple perspectives in the future.

## 5. Conclusion

In conclusion, we performed the first pan-cancer analysis of HHLA2, which indicated a substantial difference in HHLA2 expression in most tumor tissues compared to normal tissues, and revealed an association between HHLA2 expression and clinical prognosis. Moreover, we have found that the HHLA2 expression is related to the tumor microenvironment, immune cell infiltration, MSI, and TMB. Its effect on tumor immunity varies depending on the cancer type. These results contribute to shedding light on the role of HHLA2 in tumorigenesis and progression, as well as providing a new perspective on the future development of more precise and personalized immune antitumor therapies. Therefore, HHLA2 may play an important role as a prognostic biomarker across cancer and has provided new insight into the role of HHLA2 in human cancers.

## Figures and Tables

**Figure 1:** HHLA2 is abnormally expressed in human pan-cancer. (a) HHLA2 expression in 33 tumor tissues from TCGA database. (b) HHLA2 expression in diverse cancers and normal tissues from TCGA database. (c) Differential expression of HHLA2 in cancers and normal tissues from GTEx and TCGA. (d) HHLA2 expression of different tumor types in the TIMER database. The red and blue boxes represent tumor tissues and normal tissues, respectively. ∗ indicates *p* < 0.05, ∗∗ indicates *p* < 0.01, and ∗∗∗ indicates *p* < 0.001.

**Figure 2:** The effect of HHLA2 on the prognosis of various cancers using Cox proportional hazards models. (a) Forest plots showing correlations between OS and HHLA2 expression in 33 cancer types. (b) Forest plots showing correlations between DSS and HHLA2 expression in 33 cancer types. (c) Forest plots showing correlations between DFS and HHLA2 expression in 33 cancer types. (d) Forest plots showing correlations between PFI and HHLA2 expression in 33 cancer types.

The article "HHLA2 Used as a Potential Prognostic and Immunological Biomarker and Correlated with Tumor Microenvironment in Pan-Cancer" was retracted in 2024. Reasons: signs of a paper mill; suspected computer-generated content; unreliable results or conclusions; concerns about the data.

**Figure 3:** Correlation between HHLA2 expressions in patients with OS. Values of *p* < 0.05 were considered and displayed. Kaplan–Meier analyses show the association between HHLA2 expression and OS in 8 types of cancers.

**Figure 4:** Correlation between HHLA2 expressions in patients with DSS. Values of *p* < 0.05 were considered and displayed. Kaplan–Meier analyses show the association between HHLA2 expression and DSS in 7 types of cancers.

**Figure 5:** Correlation between HHLA2 expressions in patients with DFI. Values of *p* < 0.05 were considered and displayed. Kaplan–Meier analyses show the association between HHLA2 expression and DFI in 4 types of cancers.

**Figure 6:** Correlation between HHLA2 expressions in patients with PFI. Values of *p* < 0.05 were considered and displayed. Kaplan–Meier analyses show the association between HHLA2 expression and PFI in 9 types of cancers.

**Figure 7:** The correlations between mRNA HHLA2 expression and pathological stages in various cancers.

**Figure 8:** Correlation between the HHLA2 gene expression and TMB and MSI in pan-cancer. (a) A stick chart shows the correlations between HHLA2 expression and TMB in 33 types of cancers. The red curve represents the correlation coefficient, and the blue value represents the range. (b) A stick chart shows the correlation between HHLA2 and MSI in 33 types of cancers.

**Figure 9:** The HHLA2 expression correlated with the infiltration levels of various immune cells in pan-cancer.

**Figure 10:** Correlation analyses of the HHLA2 expression with immune checkpoint genes in pan-cancer.

**Figure 11:** KEGG enrichment analysis of HHLA2 in various cancers. KEGG pathways associated with HHLA2 in ACC, BRCA, COAD, HNSC, LAML, KIRC, PAAD, PRAD, and UCEC.

**Figure 12:** Correlation analyses of the HHLA2 expression with the pathway GSCA in pan-cancer. The pathway GSCA included are as follows: TSC/mTOR, RTK, RAS/MAPK, PI3K/AKT, EMT, DNA Damage Response, Cell Cycle, and Apoptosis pathways.

## Data Availability

The authors certify that all the original data in this research could be obtained from public database. The names of the repositories can be found in the article material. All data generated or analyzed during this study are included in this article.

## Supplementary Materials

Supplementary Materials Supplementary Table 1: the detailed information of 33 cancer types. Supplementary Table 2: correlation between OS and HHLA2 expression in 33 cancer types. Supplementary Table 3: correlation between DSS and HHLA2 expression in 33 cancer types. Supplementary Table 4: correlation between DFI and HHLA2 expression in 33 cancer types. Supplementary Table 5: correlation between PFI and HHLA2 expression in 33 cancer types. Supplementary Table 6: correlation between the HHLA2 gene expression and TMB in pan-cancer. Supplementary Table 7: correlation between the HHLA2 gene expression and MSI in pan-cancer. Supplementary Table 8: the HHLA2 expression correlated with the infiltration levels of various immune cells in the TIMER database. Supplementary Table 9: correlation analyses of the HHLA2 expression with immune checkpoint genes in pan-cancer. Supplementary Table 10: correlation analyses of the HHLA2 expression with the pathway GSCA in pan-cancer.
